The article "The Function of Retinal Thickness and Microvascular Alterations in the Diagnosis of Systemic Sclerosis" was retracted in 2023. Reasons: signs of a paper mill; compromised peer review; unreliable results or conclusions.

# The Function of Retinal Thickness and Microvascular Alterations in the Diagnosis of Systemic Sclerosis

**DOI:** 10.1155/2023/1805938

**Published:** 2023-02-22

**Authors:** Xia Fang, Shujiao Yu, Yilin Peng, Bozhi Huang, Min Kang, Jiangbiao Xiong, Ting Luo, Rui Wu, Yi Shao

**Affiliations:** ^1^Department of Rheumatology, The First Affiliated Hospital of Nanchang University, Nanchang, 330006 Jiangxi Province, China; ^2^Department of Ophthalmology, The First Affiliated Hospital of Nanchang University, Nanchang, 330006 Jiangxi Province, China; ^3^Jiangxi Provincial Key Laboratory of Preventive Medicine, Nanchang University, Nanchang, 330006 Jiangxi Province, China

## Abstract

In this study, we aim to investigate retinal thickness (RT) and superficial vascular density (SVD) differences between patients with systemic sclerosis (SSc) and healthy controls (HCs) by optical coherence tomography angiography (OCTA). Sixteen patients with a definitive SSc diagnosis without clinical signs of retinopathy and 16 normal control subjects were recruited. All individuals underwent OCTA scanning to assess macular RT and SVD. We divided each image into nine subregions as the early treatment diabetic retinopathy study (ETDRS). Visual acuity (VA) was considerably different between patients with SSc (32 eyes) and control subjects (32 eyes) (p < 0.001). Compared to the control group, individuals with SSc had decreased inner RT in inner superior, outer superior, outer temporal, inner temporal, center, and inner nasal regions (p < 0.05). Outer RT was decreased in the outer and inner temporal regions, and full RT was decreased in the regions of outer superior, inner superior, inner temporal, and outer temporal, in comparison to the control group (p < 0.05). Patients with SSc had significant reduction of SVD in the inner and outer of both superior and temporal, besides outer nasal regions than controls. (p < 0.05). Moreover, SVD was significantly associated with the outer temporal region of patients suffering from SSc (p < 0.05). Diagnostic Sensitivity of RT and SVD of Inner Superior Regions in SSc, as indicated by areas under curves of the Receiver Operating Characteristic (ROC), were 0.874 (95% CI: 0.786–0.962) and 0.827 (95% CI: 0.704–0.950), respectively. In conclusion, VA may be affected by RT variations inside the macula in patients with SSc. Measuring RT with OCTA could be a useful predictor of early diagnosis.

## 1. Introduction

Systemic sclerosis (SSc) is a multisystem chronic autoimmune disorder characterised by immunological activation, extensive vasculopathy, and pervasive fibrosis with diverse clinical symptoms [1, 2]. SSc is defined as substantial vascular involvement that is not restricted to the microcirculation of the skin's periphery but can also be found in the lungs, kidneys, cardiac muscles, GIT, as well as the eyes [3, 4]. Microvasculature involvement is one of the early manifestations of SSc and may contribute to severe multiorgan failure through pathological alterations, such as endothelial damage, vessel walls mononuclear cell infiltration, and obliterative lesions [5] Those structural vascular alterations, in conjunction with persistent vasospasm, may result in insufficient blood flow, tissue damage, and capillary infarction.

The article "The Function of Retinal Thickness and Microvascular Alterations in the Diagnosis of Systemic Sclerosis" was retracted in 2023. Reasons: signs of a paper mill; compromised peer review; unreliable results or conclusions.

Research papers increasingly discuss ocular symptoms among SSc patients [6, 7] and their prevalence as well as association with the underlying disease stage. The pathogenesis of ocular and related systems in patients with SSc is complicated and remains unclear [8]. The retina features microcirculation with immune privilege, a lack of adrenergic vasomotor innervation and resident fibroblasts. [9, 10] This structure appears to provide protection from SSc-related vasculopathy and fibrosis processes. However, many conflicting findings on retinal diseases in SSc have been documented in the literature. There was no correlation among SSc with retinopathy in some trials [11]. Ushiyama et al. [12] found that retinal abnormalities are frequently observed in patients with SSc (SSc 34% VS Control 8%), perhaps reflecting vascular pathological changes. Therefore, evaluation the effects of SSc on retinal disease requires additional research with a larger patient population.

Due to fact that retinal and choroidal microvasculature is clearly vulnerable to systematic vascular changes, it may provide a useful means by which to monitor disease progression in patients with SSc [13]. Because retinal tissue has the maximum oxygen extraction per blood volume, choroidal and retinal thicknesses have been proposed as prospective inflammatory predictor for autoimmune complications besides a vascular component [14]. However, research on this role for retinal thickness has been limited. OCTA is a noninvasive imaging modality that offers morphologic and quantitative data about microvascular ocular alterations. OCTA generates angiographic high-quality and slab-segmented images using the motion contrast of erythrocytes over a stationary background [4, 15] A variety of OCTA-based studies have assessed choroidal microcirculation among SSc patients and controls; however, limited data are available on retinal thickness in these groups.

To date, rare studies have used OCTA as a potential tool to assist with early diagnosis and severity evaluation in SSc. This study attempted to examine the ocular health of SSc patients and compared the RT and VD of SSc patients and normal control using OCTA.

The article "The Function of Retinal Thickness and Microvascular Alterations in the Diagnosis of Systemic Sclerosis" was retracted in 2023. Reasons: signs of a paper mill; compromised peer review; unreliable results or conclusions.

## 2. Materials and Methods

### 2.1. Subjects

This prospective cross-sectional study was conducted at the Ophthalmology and Rheumatology Department in the First Affiliated Hospital of Nanchang University (Nanchang, China) in 2021. The Rheumatology and Immunology outpatients sequentially recruited 16 patients (32 eyes) with SSc and no clinical signs of eye problems. The Centre for Ocular Diseases Clinical Research recruited healthy individuals. Data on age, sex, illness duration, autoantibody profile, and blood pressure were recorded for all subjects. Clinical examination and OCTA imaging were performed to ensure the lack of ocular abnormalities in these patients. One retina specialist assessed all patients' OTCA results with blind method.

### 2.2. Inclusion and Exclusion Criteria

SSc patients were required to satisfy the 2013 ACR/EULAR classification criteria for SSc [2]. Patients aged from 16 to 63 years without symptoms or evidence of retinal vasculitis, choroiditis, or optic neuritis were eligible to participate. In addition, hydroxychloroquine-induced chorioretinopathy was excluded for patient participation. The subsequent were further exclusion characteristics: (1) autoimmune illnesses apart from SSc; (2) systemic diseases, such as DM, grim hypertension systemic (over 179 mmHg systolic or over 109 mmHg diastolic), and ossia nerve systemic illness affecting the eyes (ossia nervus opticus); (3) choroidal or retinopathy disorder (e.g., arteriovenous disorder, glaucoma, or elevated IOP intraocular pressure); (4) history of trauma, ocular tumor, or surgery; (5) any contraindications, allergies, or local anesthesia/mydriatics intolerances; (6) complications which could impact fundus imaging; as well as (7) pregnancy or lactating women.

### 2.3. Ethical Considerations

This research complied with the Helsinki Declaration. Ethical review and approval were granted for this work by the board of Nanchang University, First Affiliated Hospital. Each participant voluntarily signed an informed consent form after reading and comprehending its contents.

### 2.4. Clinical Examinations

The following clinical tests and ocular investigations were performed for all participants: (1) immunological data as, anti-Scl-70 antibody, anti-SS-A anti-body, anti-SS-B anti-body, and ANA antibody were measured by indirect immunofluorescence assay; (2) evaluation of the patient's inflammatory status via C-reactive protein (CRP) level and erythrocyte sedimentation ratio (ESR) analyses; (3) assessment of the patient's mental state via HADS score; (4) OCTA; (5) ocular measurements, include IOP (Goldmann tonometry), VA (Snellen chart), spherical equivalent refractive error, the tear breakup time (BUT), Schirmer's test, tear meniscus height (TMH), and ocular staining score (OSS).

The article "The Function of Retinal Thickness and Microvascular Alterations in the Diagnosis of Systemic Sclerosis" was retracted in 2023. Reasons: signs of a paper mill; compromised peer review; unreliable results or conclusions.

The protocol of BUT, Schirmer's test, TMH, and OSS were examined as we have previously described [16].

BUT: fluorescein sodium was applied evenly on the ocular surface, and the first tear point film rupture was observed under cobalt blue light, and the time for this to occur was recorded. Less than 10 s was considered positive.

Schirmer's test: after disinfecting the conjunctival sac, one end of a piece of filter paper measuring (5^∗^35 mm was folded into a right angle and inserted into the conjunctival sac. Length of the wet region of the paper after 5 minutes was observed, and < 5 mm was considered positive.

TMH: this was measured under infrared light after a blink using Keratograph 5M software.

OSS: a complete evaluation was performed using corneal fluorescein staining in conjunction with conjunctival lissamine green staining. The cornea, the nasal conjunctiva, and the temporal conjunctiva were the three areas of the ocular surface that were taken into consideration for each eye. A score was given to the nasal and temporal conjunctiva based on the amount of spotty conjunctivitis in the palpebral fissure. A positive OSS index was that the score higher than or equal 3.

### 2.5. Optical Coherence Tomography Angiography

For OCTA imaging and displaying the retinal cross-section and microvasculature simultaneously, we employed system of RTVue Avanti XR (Optovue, CA). The OCTA protocol was as previously described [16]. We imaged for 3.9 seconds at a central of 840 nm wavelength and 45 nm bandwidth, while axial and horizontal resolutions were 5 mm and 22 *μ*m, respectively, all along with a scanning speed of 70,000 A scans/s. Five angiographies were captured in the mode of 3 mm^∗^3 mm scanning. In four volume scans, an overall of 933,120 A scans (2 for horizontal and vertical scans each) were obtained after four volume scans. Each eye had a 3 mm^∗^3 mm en-face OCTA angiographic imaging. Following scanning, each retinal imaging was split into nine ETDRS subregions with (0.5, 1.5, and 3 mm in radius) circles, and RT was analysed. The nine subregions include outer superior (OS), inner superior (IS), outer nasal (ON), inner nasal (IN), outer inferior (OI), inner inferior (II), outer temporal (OT), inner temporal (IT), and center (C). RT was considered as full thickness (from internal limiting membrane to retinal pigment epithelium), inner (from internal limiting membrane to inner plexiform layer) and outer (the difference between full RT and inner RT). The proportion of the region which showed vascular perfusion provided an estimate of VD, which was accomplished by generating 2D imaging en-face of superficial retina. Assign then distribute image block's value to each background (0) or perfusion (1). With the intention of calculating VD from macula centre to the edge of 3 mm × 3 mm brightness gradient image, average skeletal plate value was scaled by pixel size in the region of interest, which was 512 pixels/3 mm. We measured macular RT and SVD. In every case, we started by evaluating the subjects' right eye. The left-eye data was inverted to provide a mirror image of the right-eye data. One set of data per person was compiled by averaging the results from the left and right eyes.

The article "The Function of Retinal Thickness and Microvascular Alterations in the Diagnosis of Systemic Sclerosis" was retracted in 2023. Reasons: signs of a paper mill; compromised peer review; unreliable results or conclusions.

### 2.6. Statistical Analysis

Data were processed utilizing SPSS 24.0 and reported as mean ± standard deviation. Using RStudio and GraphPad Prism version 8, we compared independent sample groups using the t-test, chi-square, and Fisher's exact tests (La Jolla, Ca, US). All types of RTs and SVDs were compared between groups using the generalised estimation equation. Linear correlation analyses were carried out across RT groups with SVD in each group. Multiple regression models, both univariate and multivariate, were performed to determine the associations between RT and ocular factors. To analyze SVD and RT thickness groups as diagnostic indicators for SSc, Receiver Operating Characteristic (ROC) curves were plotted. Significant statistical differences were defined as those (p < 0.05). Adjustments to p values for multiple comparisons were made using a false discovery rate (FDR).

## 3. Results

### 3.1. Subjects

Mean age was similar in the control group (49.500 ± 5.955 years) and SSc group (46.750 ± 11.358 years; p = 0.398). Mean time to diagnosis for SSc patients was 3.100 ± 3.068 years. SSc patients had significantly higher HADS scores compared to controls (8.938 ± 2.839) vs. 2.813 ± 1.109; p < 0.0001) (Table 1). The SSc group exhibited lower VA (p < 0.001) and shorter BUT than the control group (5.000 ± 1.218 s vs. 13.906 ± 1.785 s; p < 0.001), lower SIT score (6.250 ± 0.762 mm vs. 12.938 ± 1.390 mm; p < 0.001) and lower TMH (0.162 ± 0.028 vs. 0.581 ± 0.123 mm; p < 0.001) (Table 2).

### 3.2. Macular RT

Table 3 and Figure 1(f) display the subregional RT for the SSc and control groups. Following age, VA, IOP, and BP adjustments, inner RT was statistically reduced in SSc patient's group than in controls in OS (p < 0.0001), IS (p < 0.001), OT (p = 0.006), IT (p = 0.033), C regions (p = 0.018), and IN region (p = 0.014) (Figure 1(c)). The remaining 3 inner retinal regions (ON, p = 0.195; II, p = 0.075; OI, p = 0.136) (Figure 1(c)) did not change significantly across groups. The outer RT in patients with SSc was statistically reduced than OT in controls (p = 0.011) and IT (p = 0.005) regions (Figure 1(d)). Full RT was statistically significant thinner in SSc than controls in IS (p = 0.019), OS (p < 0.001), IT (p = 0.001), and OT (p < 0.001) regions (Figure 1(b)). No additional differences between groups were found to be statistically significant (p > 0.05).

The article "The Function of Retinal Thickness and Microvascular Alterations in the Diagnosis of Systemic Sclerosis" was retracted in 2023. Reasons: signs of a paper mill; compromised peer review; unreliable results or conclusions.

Macular RT was strongly correlated to diastolic BP in univariate analysis (*β* = 0.176, p = 0.037) but not with VA, age, mean IOP, or systolic blood pressure. The multivariate regression analysis resulted that systolic blood pressure (*β* = −0.393, p = 0.001) was inversely correlated to macular RT. Diastolic BP (*β* = 0.347, p = 0.005) and BUT (*β* = 1.876, p = 0.044) were significantly related to thinner macular RT (Table 4).

### 3.3. Superficial Macular Retinal VD

SVD at each retinal subregions in the healthy group and SSc patients are shown in Table 5, Figures 1(a) and 1(f) following age, IOP, VA, and BP adjustments. Patients with SSc had a significantly decreased SVD than healthy subjects in the IS, OS, ON, IT, and OT regions (p ≤ 0.001) (Table 5, Figures 1(a) and 1(f)). In SSc patient's group, SVD was inversely associated to disease duration (−0.540) (Figure 2(d)).

### 3.4. ROC Curve Analysis of RT and SVD

OCTA data were analysed to assess the specificity and sensitivity of RT and SVD as diagnostic predictors of SSc-induced alterations (Figure 3). We found that IS, OS, ON, IT, and OT regions had significantly different RTs among the groups. AUC for SVD in the IS region was 0.827 (95% CI: 0.704 to 0.9500), and for the ON region, it was 0.752 (95% CI: 0.607–0.896), a diagnostic sensitivity for SVD of moderate to high for SSc (Figure 3(a)). Significant differences between groups were found in inner RT in the regions of IS, OS, IN, IT, OT, and C; outer RT in IT and OT; and full RT in IS, OS, IT, and OT. AUC for outer RT in the IS region was 0.874 (95% CI: 0.786 to 0.962), indicating moderate to high diagnostic sensitivity for SSc (Figure 3(d)).

### 3.5. Relationship between RT and SVD and Relationship between Disease Duration and HADS

SSc patients with inner RT was positively related to SVD in the OT region (r = 0.36) (Figures 2(a) and 2(b)), implying that decreased SVD is related to retinal thinning in SSc. Patients with SSc who had their condition progress over a longer period of time had increased HADS index (0.8467) (Figure 2(d)). A lower SVD was associated with longer disease duration (−0.540) in the SSc group, as we have already mentioned (Figure 2(d)).

## 4. Discussion

This study demonstrates that patients with SSc had significantly decreased VA, RT, and retinal VD, in addition to significant relationships among these parameters using OCTA. In our study, we found the SSc patients had poor visual acuity and dry eye (shorter BUT, lower SIT score and lower TMH) consistent with some previous studies. [17] Two case-control studies showed that fibrosis of the adjacent conjunctiva and lacrimal gland might induce tear production decreased in SSc [18, 19]. Moreover, they showed that SSc patients are significantly more likely to experience dry eye symptoms. In contrast to these findings, Wangkaew et al. revealed no statistical difference between SSc patients and healthy subjects after adjusting for the use of xerogenic drugs and smoking, suggesting that the utilization of drugs with anticholinergic side-effects and smoking may also be associated with higher dry eye symptom scores in SSc patients. [20, 21] Keratoconjunctivitis, skin changes of the eyelid, uveitis, episcleritis, weakening of the extraocular muscles, scleritis, glaucoma, peripheral ulcerative keratitis, enophthalmos, and cataract are some of the other clinical symptoms. One-third of SSc patients had retinal abnormalities on fundus examination, according to a cross-sectional investigation evaluating retinal involvement [12].

The article "The Function of Retinal Thickness and Microvascular Alterations in the Diagnosis of Systemic Sclerosis" was retracted in 2023. Reasons: signs of a paper mill; compromised peer review; unreliable results or conclusions.

Although its pathophysiology is poorly understood, it is widely acknowledged that SSc begins in the microcirculation network. Raynaud's phenomenon occurs at the initial stage of SSc in about 95% of patients and may guide diagnosis if accompanied by capillaroscopy abnormalities. [22, 23] Capillaroscopy is a noninvasive imaging technique that explores microcirculatory involvement and may show specific signs of the disease in patients who have Raynaud's phenomenon but no skin sclerosis. To date, capillaroscopy has been considered part of the EULAR/ACR standards for SSc and may provide useful information about prognosis for SSc patients. [2, 24] Maricq and Cutolo capillaroscopic classification system may be useful in recognizing patients at different phases of illness. [25, 26] Over time, the capillaroscopic pattern in SSc patients evolved from destruction of giant capillaries to that of capillary beds [27]. Furthermore, capillaroscopy may be used to detect a window of opportunity for treatment in patients who progress from giant capillary to capillary bed destruction. However, retinal blood vessels involved may differ qualitatively from nailfold capillaries. [12] In the evaluation of SSc, retinal vascular, ocular, and visual factors are frequently neglected. While there have been investigations looking at the choroidal and retinal vascular features in SSc [13, 28, 29], further detailed investigations at varying retinal and choroid depths using OCTA are required.

The article "The Function of Retinal Thickness and Microvascular Alterations in the Diagnosis of Systemic Sclerosis" was retracted in 2023. Reasons: signs of a paper mill; compromised peer review; unreliable results or conclusions.

Vasculopathy are the most important features of SSc, not only because they are almost always present, but also provide clues to early diagnosis, which long before the appearance of nonvascular symptoms. [22, 23] Because retinal vasculature indicates systemic arteriolar and capillary pathology in SSc, early diagnosis of ocular microcirculation involvement is crucial. The different layers of retina acquire nutrition from different vessel: outer layer acquire from choroidal vessels, the inner layer acquire from the central retinal blood vessels, and the macular region acquire from choroidal capillaries. The posterior eye is one of the tissues in the body that has the highest metabolic activity. As a consequence, it is exceedingly vulnerable to capillary injury [30, 31]. Once the vasculopathy happened in the retina, the pathology of the retinal region will also be changed, which might affect the whole choroidal and retinal vascular network. Our research revealed that the retinal SVD is significantly diminished in all layers among SSc patients. The thickness of the inner RT had a positive correlation with the SVD (Figure 4). Studies have found the changes of microcirculation may develop long before clinically detectable retinopathy. Similarly, we speculate that subclinical alteration also exists in SSc patients.

SSc mainly targets small arteries and capillaries by decreasing their density and obliterating them. [32] The retinal and choroidal vasculature would be perfect for observing pervasive arteriolar and capillary pathology in SSc, making the early diagnosis of changes to ocular microcirculation crucial. Rommel et al. [13] found in SSc group that the perfusion of the retinal and choroidal was significantly decreased. This suggests that retinal or choroidal perfusion is involved in early stages of the disease and eventually impacts vascular dysfunction in both tissues, suggesting that retinal and choroidal examinations should be considered immediately after SSc diagnosis to detect early alterations. In our research, RT was found to be lowered in all retinal regions of SSc patients by ETDRS partition method, including the IS, OS as well as IT area of inner retina and OT and IT area of outer retina, in addition to OT and IT area of full-thickness retina. To our knowledge, this is first report of retinal thickness evaluation in SSc using OCTA.

Our investigation of the ROC curve for SVD and inner RT in the IS region revealed a potential diagnosis method for early detection of retinal alterations in SSc. Early diagnosis and evaluation are essential for effective therapy and a favourable prognosis. SSc is a heterogeneous disease that may progress to fatal complications after several months or may remain limited to sclerodactyly and Raynaud's phenomenon. The detection of an increased risk of complications in scleroderma is important to recognize patients at risk of progression to severe complications. OCTA is a noninvasive and an easy technology that offers information on the perfusion of the intraocular vascular network. Alteration in microcirculation may precede clinically retinopathy in people with SSc; hence, OCTA is a good approach for distinguishing healthy eyes from those affected by SSc.

The article "The Function of Retinal Thickness and Microvascular Alterations in the Diagnosis of Systemic Sclerosis" was retracted in 2023. Reasons: signs of a paper mill; compromised peer review; unreliable results or conclusions.

The RT assessed by OCTA may aid in the imaging diagnosis of SSc, however additional research is required for future clinical application. Given the importance of this study's findings, more analyses of data from a larger number of participants with greater clinical diversity will be required to confirm our findings. Moreover, we should differentiate the patient suffered from limited form of SSc or diffused form of SSc, which showed different severity, clinical manifestations, complications, prognosis, and survival.

## 5. Conclusion

We utilised OCTA to improve our understanding of RT and SVD in SSc patients. The results suggested that the inner, outer, and total RT were thinner in SSc patients, whereas the SVD was reduced in the IS, OS, ON, OT, and IT regions. In addition, a positive correlation was detected between changes in RT and SVD. Thus, OCTA may aid in the imaging-assisted diagnosis of SSc.

## Figures and Tables

**Figure 1:** The RT and SVD analyses and OCTA images. (a) Regional analysis of SVD in the SSc and control groups. The vertical coordinate is SVD value; the horizontal coordinate is retinal subregions. (b–d) Regional analysis of three types of RT between SSc and control groups. The vertical axis represents RT values, whereas the horizontal axis represents retinal regions. (e) RT in a cross-sectional OCTA study of SSc and control group. ETDRS was used to evaluate the inner, full RT, and SVD. (f) Comparing the SSc and control groups in the nine subregions of SVD and three types of RT. ∗, p < 0.05; ∗∗, p < 0.01; ∗∗∗, p < 0.001; ∗∗∗∗, p < 0.0001.

**Figure 2:** Relationship between RT and SVD in SSc patients and healthy controls and association between disease duration and both HADS and SVD. (a and b) In patients with SSc, SVD was actively linked to inner RT in the OT region (r = 0.36; p = 0.043). (c) A significant correlation was found between disease duration and HADS (r = 0.8457, p < 0.0001). (d) Disease duration was inversely related to SVD in the region of OT. (r = −0.540, p = 0.0309).

**Figure 3:** ROC curve analysis of RT and SVD. (a) The area under the ROC curve for SVD was 0.827 (95% CI: 0.704 to 0.9500) in IS, 0.827 in OS (95% CI: 0.704 to 0.950), 0.734 in ON (95% CI: 0.607 to 0.862), 0.701 in IT (95% CI: 0.564 to 0.837), and 0.720 in OT (95% CI: 0.583−0.856). (b) The area under the ROC curve for outer RT was 0.777 (95% CI: 0.656 to 0.899) for IT and 0.750 for OT (95% CI: 0.619 to 0.880). (c) The area under the ROC curve for full RT was 0.701 (95% CI: 0.569 to 0.833) for IS, 0.779 for OS (95% CI: 0.666 to 0.892), 0.774 for IT (95% CI: 0.654 to 0.894), and 0.784 for OT (95% CI: 0.669−0.900). (d) The area under the ROC curve for inner RT was 0.874 (95% CI: 0.786 to 0.962) for IS, 0.768 for Inner OS (95% CI: 0.648−0.888), 0.695 for IN (95% CI: 0.648 to 0.888), 0.678 for IT (95% CI: 0.540−0.816), 0.693 for OT (95% CI: 0.565 to 0.822), and 0.675 for C (95% CI: 0.536−0.813).

The article "The Function of Retinal Thickness and Microvascular Alterations in the Diagnosis of Systemic Sclerosis" was retracted in 2023. Reasons: signs of a paper mill; compromised peer review; unreliable results or conclusions.

**Figure 4:** Relationship between SVD, RT, and visual in SSc patient. The decrease of superficial retinal vascular density might induce related area of retinal thickness decreased, and then resulted poorer vision at last.

**Table 1:** Demographic and clinical data from SSc patients and normal controls.

	SSc (n = 16, 32 eyes)	Control (n = 16, 32 eyes)	p value
Age (y)	46.750 ± 11.358	49.500 ± 5.955	0.398^a^
Gender			
Female	12	14	0.654^b^
Duration of SSc (y)	3.100 ± 3.068	N/A	
ESR (mm/h)	23.484 ± 22.497	N/A	
CRP (10 mg/L)	4.723 ± 4.720	N/A	
ANA, n (%)	13 (81.250)	N/A	
Scl-70), n (%)	6 (37.500)	N/A	
Anti SSA/Ro, n (%)	4 (25.000)	N/A	
Anti SSB/La, n (%)	0 (0.000)	N/A	
Systolic blood pressure (mm Hg)	112.813 ± 14.625	124.438 ± 5.738	0.0060^a^
Diastolic blood pressure (mm Hg)	72.875 ± 13.386	82.938 ± 6.298	0.0107^a^
HADS	8.938 ± 2.839	2.813 ± 1.109	**< 0.0001** ^**a**^

Note: bold values indicate p < 0.05; ^a^independent t test; ^b^ chi-square test. Abbreviations: ANA: antinuclear antibody; anti-topo I (Scl-70): anti-DNA topoisomerase I; N/A: not applicable.

**Table 2:** Ocular and visual data from patients with SSc and healthy controls.

	SSc (n = 16, 32 eyes)	Control (n = 16, 32 eyes)	p value^a^
VA (logMAR)	0.644 ± 0.254	0.9 ± 0.134	< **0.001**
Mean IOP (mm Hg)	15.656 ± 1.865	15.225 ± 1.689	**0.426**
BUT (s)	5.000 ± 1.218	13.906 ± 1.785	< **0.001**
SIT (mm)	6.250 ± 0.762	12.938 ± 1.390	< **0.001**
TMH (mm)	0.162 ± 0.028	0.581 ± 0.123	< **0.001**

Note: bold values indicate p < 0.05. ^a^p value was obtained using a generalized estimation equation (data from both eyes were included).

**Table 3:** Regional macular RT compared across patients with SSc and normal controls.

Location	SSc (n = 16, 32 eyes)	Control (n = 16, 32 eyes)	p value	FDR^a^
Macular inner retinal thickness (*μ*m, mean ± SD)				
IS	104.781 ± 6.494	113.781 ± 5.482	< 0.001	**< 0.001**
OS	103.219 ± 8.385	111.000 ± 5.853	< 0.001	**< 0.0001**
IN	111.781 ± 6.514	115.781 ± 5.802	0.022	**0.014**
ON	122.531 ± 7.229	123.469 ± 4.280	0.610	0.195
II	112.156 ± 6.222	114.344 ± 5.445	0.204	0.075
OI	103.188 ± 6.963	104.813 ± 6.463	0.396	0.136
IT	101.844 ± 6.461	104.438 ± 4.614	0.078	**0.033**
OT	90.938 ± 5.465	94.781 ± 5.110	0.006	**0.006**
C	48.938 ± 6.283	52.344 ± 5.463	0.036	**0.018**
Macular outer retinal thickness (*μ*m, mean ± SD)				
IS	218.906 ± 15.378	216.781 ± 5.723	0.533	0.708
OS	188.500 ± 12.083	193.250 ± 12.746	0.139	0.386
IN	217.813 ± 11.616	218.406 ± 12.745	0.863	0.797
ON	195.219 ± 15.737	195.063 ± 8.583	0.969	0.815
II	211.406 ± 13.671	211.813 ± 7.046	0.900	0.804
OI	180.969 ± 10.811	180.469 ± 12.959	0.876	0.799
IT	206.875 ± 7.606	214.094 ± 8.216	0.001	**0.005**
OT	179.344 ± 6.302	187.063 ± 10.895	0.003	**0.011**
C	192.594 ± 25.615	194.469 ± 15.046	0.691	0.758
Macular full retinal thickness (*μ*m, mean ± SD)				
IS	323.688 ± 11.828	330.563 ± 7.746	0.016	**0.019**
OS	291.719 ± 11.450	304.250 ± 11.992	< 0.001	**< 0.001**
IN	329.594 ± 11.092	334.188 ± 15.135	0.212	0.198
ON	317.750 ± 11.144	318.531 ± 8.944	0.791	0.437
II	323.563 ± 10.485	326.156 ± 9.354	0.386	0.305
OI	284.156 ± 9.792	285.281 ± 13.187	0.708	0.446
IT	308.719 ± 12.822	318.531 ± 7.431	0.001	**0.001**
OT	270.281 ± 8.862	281.844 ± 11.043	< 0.001	**< 0.001**
C	241.531 ± 28.778	246.813 ± 16.585	0.312	0.216

Note: bold values indicate p < 0.05. ^a^ Generalized estimation equation models were applied to attain p values comparing mean inner, outer as well as full macular RT in SSc patients and healthy subjects. Models were adjusted for age, IOP, VA, and BP.

The article "The Function of Retinal Thickness and Microvascular Alterations in the Diagnosis of Systemic Sclerosis" was retracted in 2023. Reasons: signs of a paper mill; compromised peer review; unreliable results or conclusions.

**Table 4:** Macular RT and its correlation with demographic and ocular parameters in patients with SSc: a univariate and multivariate regression analyses.

Parameters	Univariate regression analysis regression coefficient (*β* ± SE)	p value^a^	Multivariate regression analysis Regression coefficient (*β* ± SE)	p value^a^
Age (y)	−0.008 ± 0.103	0.941	−0.127 ± 0.094	0.270
VA (logMAR)	0.094 ± 4.518	0.984	5.883 ± 4.299	0.368
Mean IOP (mm Hg)	0.038 ± 0.615	0.951	0.876 ± 0.618	0.310
Systolic blood pressure (mm Hg)	0.112 ± 0.076	0.155	−0.393 ± 0.106	**0.001**
Diastolic blood pressure (mm Hg)	0.176 ± 0.081	**0.037**	0.347 ± 0.111	**0.005**
BUTs	0.522 ± 0.937	0.582	1.876 ± 0.881	**0.044**
SIT (mm)	0.194 ± 1.505	0.898	−1.867 ± 1.189	0.129

Note: bold values indicate p < 0.05. ^a^p value was obtained with generalized estimating equation.

**Table 5:** Regional SVD compared in patients with SSc and normal controls.

Region (%, mean ± SD)	SSc (n = 16, 32 eyes)	Control (n = 16, 32 eyes)	p value	FDR^a^
IS	44.656 ± 9.472	53.438 ± 3.877	< 0.001	**< 0.001**
OS	45.281 ± 8.379	50.875 ± 3.319	0.001	**< 0.001**
IN	49.406 ± 11.736	51.031 ± 3.524	0.456	0.105
ON	48.344 ± 7.698	53.969 ± 2.788	< 0.001	<0.001
II	51.188 ± 7.643	52.688 ± 3.596	0.291	0.073
OI	50.188 ± 7.235	52.313 ± 3.856	0.105	0.052
IT	46.250 ± 10.887	53.406 ± 4.482	0.001	**0.001**
OT	45.188 ± 7.204	50.250 ± 3.379	0.002	**0.001**
C	25.781 ± 10.354	27.781 ± 5.482	0.349	0.082

Note: bold values indicate p < 0.05. ^a^ Mean SVD was compared between Healthy and SSc patients using generalised estimating equation models, and p values were calculated.

The article "The Function of Retinal Thickness and Microvascular Alterations in the Diagnosis of Systemic Sclerosis" was retracted in 2023. Reasons: signs of a paper mill; compromised peer review; unreliable results or conclusions.

## Data Availability

The data used to support the findings of this study are included within the article.

## References

[1] Bobeica C., Niculet E., Musat C. L. (2022). Paraclinical aspects in systemic sclerosis. *International Journal of General Medicine*.

[2] van den Hoogen F., Khanna D., Fransen J. (2013). 2013 classification criteria for systemic sclerosis: an American college of rheumatology/European league against rheumatism collaborative initiative. *Arthritis & Rheumatism*.

[3] Allanore Y., Simms R., Distler O. (2015). Systemic sclerosis. *Nature Reviews. Disease Primers*.

[4] Rothe M., Rommel F., Klapa S. (2019). Evaluation of retinal microvascular perfusion in systemic sclerosis: a case-control study. *Annals of the Rheumatic Diseases*.

[5] Gabrielli A., Avvedimento E., Krieg T. (2009). Scleroderma. *The New England Journal of Medicine*.

[6] Schwaiger J., Loder C. D., Dobarro D. (2017). Optical coherence tomography evaluation of pulmonary arterial vasculopathy in systemic sclerosis. *Scientific Reports*.

[7] Carnevali A., Giannaccare G., Gatti V. (2021). Retinal microcirculation abnormalities in patients with systemic sclerosis: an explorative optical coherence tomography angiography study. *Rheumatology (Oxford, England)*.

[8] Kozikowska M., Luboń W., Kucharz E., Mrukwa-Kominek E. (2020). Ocular manifestations in patients with systemic sclerosis. *Reumatologia*.

[9] Aissopou E., Bournia V. K., Protogerou A. D. (2015). Intact calibers of retinal vessels in patients with systemic sclerosis. *The Journal of Rheumatology*.

[10] Streilein J. (2003). Ocular immune privilege: therapeutic opportunities from an experiment of nature. *Nature Reviews Immunology*.

[11] Grennan D., Forrester J. (1977). Involvement of the eye in SLE and scleroderma. A study using fluorescein angiography in addition to clinical ophthalmic assessment. *Annals of the Rheumatic Diseases*.

[12] Ushiyama O., Ushiyama K., Yamada T. (2003). Retinal findings in systemic sclerosis: a comparison with nailfold capillaroscopic patterns. *Annals of the Rheumatic Diseases*.

The article "The Function of Retinal Thickness and Microvascular Alterations in the Diagnosis of Systemic Sclerosis" was retracted in 2023. Reasons: signs of a paper mill; compromised peer review; unreliable results or conclusions.

[13] Rommel F., Prangel D., Prasuhn M., Grisanti S., Ranjbar M. (2021). Correlation of retinal and choroidal microvascular impairment in systemic sclerosis. *Orphanet Journal of Rare Diseases*.

[14] Steiner M., Esteban-Ortega M., Muñoz-Fernández S. (2019). Choroidal and retinal thickness in systemic autoimmune and inflammatory diseases: a review. *Survey of Ophthalmology*.

[15] Rommel F., Siegfried F., Sochurek J. A. M. (2019). Mapping diurnal variations in choroidal sublayer perfusion in patients with idiopathic epiretinal membrane: an optical coherence tomography angiography study. *International Journal of Retina and Vitreous*.

[16] Liu R., Wang Y., Li Q. (2022). Optical coherence tomography angiography biomarkers of retinal thickness and microvascular alterations in Sjogren's syndrome. *Frontiers in Neurology*.

[17] Gomes B. A., Santhiago M. R., Magalhães P., Kara-Junior N., de Azevedo M. N., Moraes H. V. (2011). Ocular findings in patients with systemic sclerosis. *Clinics*.

[18] Sahin Atik S., Koc F., Akin Sari S., Sefi Yurdakul N., Ozmen M., Akar S. (2016). Anterior segment parameters and eyelids in systemic sclerosis. *International Ophthalmology*.

[19] Wangkaew S., Kasitanon N., Sivasomboon C., Wichainun R., Sukitawut W., Louthrenoo W. (2006). Sicca symptoms in Thai patients with rheumatoid arthritis, systemic lupus erythematosus and scleroderma: a comparison with age-matched controls and correlation with disease variables. *Asian Pacific Journal of Allergy and Immunology*.

[20] Tariq M., Amin H., Ahmed B., Ali U., Mohiuddin A. (2022). Association of dry eye disease with smoking: a systematic review and meta-analysis. *Indian Journal of Ophthalmology*.

[21] Swaminathan S., Goldblatt F., Dugar M., Gordon T. P., Roberts-Thomson P. J., South Australian Cohort (2008). Prevalence of sicca symptoms in a South Australian cohort with systemic sclerosis. *Internal Medicine Journal*.

[22] Hughes M., Allanore Y., Chung L., Pauling J. D., Denton C. P., Matucci-Cerinic M. (2020). Raynaud phenomenon and digital ulcers in systemic sclerosis. *Nature Reviews Rheumatology*.

[23] Cutolo M., Soldano S., Smith V. (2019). Pathophysiology of systemic sclerosis: current understanding and new insights. *Expert Review of Clinical Immunology*.

[24] Boulon C., Aiouaz S., Blaise S. (2019). Correlation between capillaroscopic classifications and severity in systemic sclerosis: results from SCLEROCAP study at inclusion. *Clinical and Experimental Rheumatology*.

[25] Cutolo M., Sulli A., Pizzorni C., Accardo S. (2000). Nailfold videocapillaroscopy assessment of microvascular damage in systemic sclerosis. *The Journal of Rheumatology*.

[26] Maricq H., Harper F. E., Khan M. M., Tan E. M., LeRoy E. (1983). Microvascular abnormalities as possible predictors of disease subsets in Raynaud phenomenon and early connective tissue disease. *Clinical and Experimental Rheumatology*.

The article "The Function of Retinal Thickness and Microvascular Alterations in the Diagnosis of Systemic Sclerosis" was retracted in 2023. Reasons: signs of a paper mill; compromised peer review; unreliable results or conclusions.

[27] Gheorghiu A., Oneata R., Ancuta I. (2020). Capillary loss reflects disease activity and prognosis in patients with systemic sclerosis. *Experimental and Therapeutic Medicine*.

[28] Kılınç Hekimsoy H., Şekeroğlu M. A., Koçer A. M., Akdoğan A. (2020). Analysis of retinal and choroidal microvasculature in systemic sclerosis: an optical coherence tomography angiography study. *Eye (London, England)*.

[29] Ranjbar M., Rothe M., Klapa S. (2020). Evaluation of choroidal substructure perfusion in patients affected by systemic sclerosis: an optical coherence tomography angiography study. *Scandinavian Journal of Rheumatology*.

[30] Kök M., Ayan A., Fatih Küçük M., Erol M. K., Yaprak L. (2021). Evaluation of the direct effects on retinal and choroidal microvascularity of systemic scleroderma. *Microvascular Research*.

[31] Takayama K., Kaneko H., Ito Y. (2018). Novel classification of early-stage systemic hypertensive changes in human retina based on OCTA measurement of choriocapillaris. *Scientific Reports*.

[32] Sakkas L. (2005). New developments in the pathogenesis of systemic sclerosis. *Autoimmunity*.

